# Recent Trends in Detection of Huntingtin and Preclinical Models of Huntington's Disease

**DOI:** 10.1155/2014/190976

**Published:** 2014-05-14

**Authors:** Neelima Mantha, Nandita G. Das, Sudip K. Das

**Affiliations:** Department of Pharmaceutical Sciences, Butler University, 4600 Sunset Avenue, Indianapolis, IN 46208, USA

## Abstract

Huntington's disease is a genetically inherited neurodegenerative disease that is characterized by neuronal cell death in the brain. Molecular biology techniques to detect and quantify huntingtin protein in biological samples involve fluorescence imaging, western blotting, and PCR. Modified cell lines are widely used as models for Huntington's disease for preclinical screening of drugs to study their ability to suppress the expression of huntingtin. Although worm and fly species have been experimented on as models for Huntington's disease, the most successful animal models have been reported to be primates. This review critically analyses the molecular biology techniques for detection and quantitation of huntingtin and evaluates the various animal species for use as models for Huntington's disease.

## 1. Introduction

Huntington's disease (HD) is a genetically inherited neurodegenerative disease that is characterized by neuronal cell death in the brain. The symptoms of the disease include progressive loss of cognition, balance, and mobility. The cause of HD has been identified as a mutation in the gene coding for the protein huntingtin (Htt). Htt is a ubiquitous protein occurring in both the central nervous system and peripheral tissues, with the highest levels occurring in the brain. Htt is a large protein comprising of about 3144 amino acids that has a polyglutamine (polyQ) tract in the exon-1 at the N-terminal end. In normal individuals, the numbers of glutamines range from 6 to 35 [1]. Mutation in the gene leads to an increase in the number of glutamines in the polyQ tract, because of which the number of glutamines can range from 37 to 200 in affected individuals. Although the definite functions of the Htt protein are not clear, researchers observe that it plays important roles in transcription and cytoskeletal stability. At the cellular level, the change in protein structure also disrupts the functionality of the various transcription factors [2].

## 2. Methods for Identification and Quantitation of Htt Protein

In vitro and in vivo models are valuable tools for gaining insight into the pathophysiology of HD and eventually for the development of potential cures. The development and selection of an appropriate model for the disease are a vital step in the experimental design. The quantitation of the mutant Htt protein is the critical end point to establish a disease model and to determine the efficacy of experimental drugs. A brief overview of the identification and quantitation methods for Htt protein is given below.

### 2.1. Quantitation by Fluorescence

In a HD model, if a fluorescent reporter gene is introduced in conjunction with the Htt gene, it can facilitate the detection of the Htt protein. In most cases, the intensity of the fluorescent signal can be directly correlated with the quantity of Htt protein produced. The studies performed by Kazantsev et al. were one of the early studies that reported the identification of mutant Htt aggregates with the help of enhanced green fluorescent protein (EGFP). They assayed polyQ aggregation in an array of cell lines including COS-1, COS-7, HeLa, and PC-12 cells. In the representative images of assayed COS-1 cells, fluorescence clearly differentiated between normal length of polyQ tract (25 Q) and mutant polyQ tract (104 Q). According to Kazantsev et al.'s findings, the Htt with normal polyQ length showed a diffuse cytoplasmic presence whereas the mutant Htt with a 104 Q tract showed multiple aggregates in both the nucleus and cytoplasm [3].

In their studies of an in vitro model of HD, Liu et al. incorporated EGFP as a reporter gene in COS-7 that expressed the exon-1 part of Htt gene. The COS-7 cells produced either a wild-type Htt protein with a polyQ length of 17 Q or a mutant Htt protein with a polyQ length of 72 Q. When observed under a fluorescence microscope, representative images clearly differentiated between normal sized Htt protein and the mutant Htt EGFP aggregates [4].

Aiken et al. used an inducible PC-12 cell line as an in vitro model in their studies on cell-based screening for HD drugs. Tebufenozide was the inducer and the cells produced exon-1 of the mutant Htt protein with a 103 Q polyQ tract fused with EGFP. Their results show that, following treatment with Tebufenozide, there is a progressive accumulation of Htt protein aggregates as shown by fluorescence images over a period of 72 hours. In this case, the cells not treated with the inducer acted as the control [5]. The fluorescence method of determining mutant Htt aggregates was also reported in other studies using PC-12 cells expressing wild-type and mutant Htt. Scotter et al., in their studies in PC-12 cells, further extended the utility of identification via fluorescence reporters. They described three methods, namely, find spots, granularity, and cell scoring assays to quantitate the fluorescent signal emitted by the mutant aggregates [6]. Thus, quantitation by fluorescence methods has proven to be fast and efficient for the identification and quantitation of mutant Htt protein production across a wide range of cell culture models.

### 2.2. Quantitation by Western Blotting

Western blotting or immunoblotting is an established analytical technique for the detection of specific proteins and their relative quantitation. Western blotting has the distinct advantage of specificity over other methods of detection. It also has the versatility of being a robust test in a variety of in vitro and in vivo HD models. Several studies have reported on the use of western blots for the identification and quantitation of Htt protein. The type of gels used for separation, the antibodies used, and specific protocol modifications were optimized by individual researchers according to the type of cell line and length of mutant Htt protein. An in vitro model for HD was developed by S. H. Li and X. J. Li in PC-12 cells where the cells were transfected with a plasmid coding for the exon-1 part of the Htt gene with a polyQ tract of 150 Q. In the cells used as controls, the length of the polyQ tract was 20 Q. Stably transfected cell lines were selected using Geneticin (G 418), and the researchers used western blotting to establish that the N-terminal mutant Htt protein was being produced by the transfected cells. Total protein was extracted from the cells and resolved on a polyacrylamide gel (8–12%), detected with Htt specific primary antibody EM48, and visualized using a chemiluminescence (ECL) kit. The western blotting procedure successfully established the production of mutant Htt protein from the stably transfected cells [7].

Wang et al. developed an inducible PC-12 cell line as an in vitro model for HD and used western blotting to establish the production of the mutant Htt protein. The PC-12 cells were transfected with a plasmid coding for the first 63 amino acids of the Htt protein with a polyQ tract of length 148 Q. The PC-12 cells with the normal Htt sequence produced a polyQ tract of length 23 Q. The Htt protein was tagged with myc at its C-terminal end. The cells were maintained in a culture medium that contained doxycycline, and mutant protein production was induced when doxycycline was removed from the culture medium. The cells were lysed and total protein was extracted and resolved on 4–15% gradient polyacrylamide gels. Following transfer to a nitrocellulose membrane, mutant Htt protein was identified using a primary antibody against C-terminal myc and visualized by chemiluminescence using ECL kit. The western blotting studies successfully established the production of mutant Htt protein from the inducible cells [8].

Wang et al. identified and quantitated mutant Htt protein by western blotting both in vitro in COS-7 cells and in vivo from the striatum of mice brain following treatment with siRNA. Following standard cell lysis procedures, the lysates were loaded onto gradient 5–10% SDS-polyacrylamide gels and transferred to Immobilon-P membranes after resolution. The membranes were incubated with primary antibody against Htt protein (MAB 5374) and visualized in a chemiimager. The western blotting approach was successful in quantifying the levels of mutant Htt protein in the control as well as siRNA treatment groups [9].

The studies described thus far identified mutant Htt protein by using antibodies that were targeted to a part of the Htt protein. However, the levels of Htt protein and the presence of mutant protein can also be monitored indirectly by means of proteins that interact with the Htt protein. Such proteins are called huntingtin interacting proteins (HIPs). The levels of HIPs, as well as a change in their levels, directly correlate to a change in Htt levels. The studies of interactions between Htt and various HIPs have proven valuable in determining the physiological role of the Htt protein and its effect on cellular processes consequent to the mutation. In their studies involving the interaction between transcription factor Sp1 and Htt protein, Qiu et al. used the western blotting technique to monitor the levels of Sp1 and mutant Htt to determine possible interactions between the two proteins. They studied the effects of knocking down Sp1 protein on the levels of mutant Htt both in vitro in PC-12 cells and in vivo in transgenic R6/2 HD mice. Following the knockdown of Sp1, the cells were lysed and the levels of mutant Htt were measured in untreated and treated groups. After transfer onto nitrocellulose, the membranes were treated with polyclonal antibodies that react with both polyQ tract and Sp1. Their results showed an interaction between Sp1 and mutant Htt and that the levels of mutant Htt decreased in the Sp1 knockout groups [10].

As shown in the studies above, the detection and quantitation of Htt protein by western blotting are proven effective. However, the method must be optimized for process variables such as the viscosity of the gel, run time, buffer concentration, type of membrane, time for membrane transfer and capacity, type of molecular weight ladder, and most importantly the type of primary antibody. The choice of the antibody varies based on the nature of the mutant Htt produced and the presence of any reporter genes. Hence, despite the fact that western blotting principles are well established, care should be taken to develop a robust protocol that would yield reproducible results. A recent study reported detection of variations of HTT levels in blood samples using an ELISA method. In addition, the ELISA method could differentiate between peripheral cells isolated from healthy volunteers and HD patients at different disease stages [11].

### 2.3. Quantitation by Polymerase Chain Reaction

Polymerase chain reaction (PCR) is a technique by which a particular DNA sequence can be amplified and quantitated. Reverse transcriptase PCR is a variant of PCR, in which a particular RNA is reverse-transcribed to DNA and then amplified. Thus, Htt mRNA can be reverse-transcribed and the levels of cDNA can be measured. The levels of Htt mRNA directly correlate to the levels of Htt protein in the neuronal cells. qPCR can be used to establish the production of Htt protein or to evaluate gene knockdown after treatment with potential therapeutic moieties. In in vivo studies involving a rat model for HD, Franich et al. used adeno-associated viral (AAV) vectors to introduce N-terminal mutant Htt constructs with a 70 Q polyQ tract into rat brains. Following the introduction of the mutant constructs, they used a qPCR method for the detection of Htt constructs in the striatum of the rat brains. Their results demonstrated more than a 100-fold increase in Htt levels in comparison to endogenous Htt levels, and this was successfully quantitated by qPCR [12].

In studies involving an in vitro model for HD in COS-7 cells, Liu et al. used qPCR to study the knockdown of mutant Htt gene following treatment with siRNA. Their results demonstrated an 80% decrease in the levels of Htt mRNA between the siRNA treated and untreated groups when normalized against the housekeeping genes *β*-actin and GAPDH. Thus, qPCR was successful in quantifying the relative levels of Htt mRNA and thus Htt protein, between different treatment groups [4]. Also, droplet digital PCR (ddPCR) was used to quantify human HTT messenger RNA and discriminate between the mutant and wild-type HTT alleles [13].

## 3. Models of Huntington's Disease

The majority ofHD disease models have been engineered to produce mutant Htt protein, and it is interesting to note that the mutant Htt protein in its full length or in its truncated (exon-1) form produces HD pathology both in vitro and in vivo.

### 3.1. In Vitro Models of Huntington's Disease

Since the Htt protein is amenable to being engineered with variable polyQ lengths in a variety of cell lines, such HD models provide an excellent platform to gain better insight into the disease pathogenesis and to explore treatment options. In vitro models of HD are developed by the introduction of a plasmid that encodes the mutant Htt protein into a number of mammalian cell lines. Additionally a reporter gene such as the green fluorescent protein or red fluorescent protein is routinely engineered into the plasmid for convenient detection via imaging. In the in vitro models, the hallmark of HD pathology is the formation of nuclear mutant Htt protein aggregates in the form of neuronal inclusions. In addition, there is an increase in cell motility due to apoptosis.  Table 1 describes the in vitro HD models developed using various cell lines.

### 3.2. In Vivo Models of Huntington's Disease

In vivo models for HD have been developed in a number of organisms including the ringworm* Caenorhabditis elegans*,* Drosophila*, mice, and rats. In the lower animal models, there is no sequence homology in the Htt protein with that of human Htt. However, following the discovery of the Htt sequence, rodent models were developed to express N-terminal Htt or full-length human Htt. In their review, van Raamsdonk et al. present the existing in vivo HD models and describe how they correlate to the spectrum of HD symptoms in humans [18]. Their compilation of HD models is reproduced in Table 2.

As can be seen in Table 2, the lower animal models cannot reproduce motor and cognitive deficits; therefore, they can serve as simple platforms for initial drug screening but not for detailed analyses. The higher rodent models are a good match for therapeutic efficacy trials and proof of principle studies. Among the mice models, the R6/2 and R6/1 models are well established with many research articles referring to work done using these models. These models have a mutant Htt with a polyQ tract of greater than 100, and they replicate the behavioral and motor dysfunctions adequately. In addition, they undergo significant loss of brain tissue within a short period, thus serving as excellent models for studying HD [19]. A recent study reported the development of a humanized mouse model Hu97/18 that lacks the mouse homolog but has one human muHTT gene and one human wtHTT gene, thus making it genetically equivalent to human HD patients [20].

## 4. Symptomatic Relief of Huntington's Disease Symptoms in Animal Models

In addition to histochemical tests, researchers have examined the cross-sections of the affected brain to assess loss in brain tissue and the physiological response to potential treatments. The symptomatic relief tests are performed in animal models following treatment with potential therapeutic moieties. In the studies of a R6/2 mouse model of HD, Wang et al. performed the rotarod test to determine the effect of siRNA treatment on the affected mice. The time taken for the mice to clasp their feet while hanging varied significantly among the wild-type, untreated, and treated groups. They also recorded a difference in body weight between groups with and without treatment [9].

DiFiglia et al. also reported an improvement in motor functions of R6/2 mice expressing N-terminal mutant Htt fragments following a single intrastriatal injection of cholesterol conjugated siRNA [21]. In a rat model for HD, Franich et al. determined the change in motor functions and balance as a symptomatic marker for the expression of mutant Htt in rat brains [12]. Thus, the symptomatic studies in animal models are of great value in determining efficacy of treatments or to confirm disease pathogenesis.

## 5. Conclusions

Both in vitro and in vivo experimental models of HD are invaluable for understanding disease pathogenesis, in screening the potential drugs, and in determining the efficacy of lead molecules. The biochemical methods described in this paper are well established for the analysis of Htt protein in in vitro cell lines and in vivo tissues. The symptomatic relief studies performed in higher animal models are proof of principle studies affirming the results obtained in the biochemical analytical studies.

## Figures and Tables

**Table 1:** In vitro Huntington's disease models.

Cell line	Number of glutamines in the polyQ tract	Full- length/truncated mutant protein	Reporter	Reference
HEK-293	82	N-Terminal part of Htt protein with 171 amino acids	None	[14]

HeLa A 459 Sh-SY5Y	128	N-Terminal part of Htt protein with 171 amino acids	Enhanced green fluorescent protein	[15]

Cos-7 SH-SY5Y neuro-2A	49, 72, 151	Full length of exon-1	Enhanced green fluorescent protein	[4]

HEK 293	60, 150	N-Terminal part of exon-1	Enhanced green fluorescent protein	[16]

PC-12	103	N-Terminal part of exon-1	Ecdysone inducible system	[17]

HEK 293 PC-12	150	N-Terminal part of exon-1	None	[7]

**Table 2:** Preclinical models of Huntington's disease (reproduced with permission from van Raamsdonk et al. [18]).

Human HD symptoms	Cell models	Worm models	Fly models	Neurotoxin models (mouse/rat/monkey)	N-Terminal models (mouse/rat)	Knock in mouse models	Full-length mouse models
Motor deficits	n/a	Yes	Yes	Yes	Yes	Yes	Yes
Cognitive impairment	n/a	n/a	n/a	Yes	Yes	No	Yes
Atrophy	Yes	n/a	n/a	Yes (selective)	Yes	Yes (selective)	Yes (selective)
Neuronal loss	Yes	No	Yes	Yes (selective)	Yes/no	No	Yes (selective)
Progressive phenotype	n/a	No	Yes	No	Yes	Yes	Yes
Full-length mutant Htt	Yes/no	No	Yes/no	No	No	Yes	Yes
Studies of pathogenesis	Yes	Yes	Yes	No	Yes	Yes	Yes
Screening assays for therapeutic compounds	Yes	Yes	Yes	Yes	No	No	No
Therapeutic trials	No	No	No	Yes	Yes	No	Yes
